# Resolution of Joint Molecules by RuvABC and RecG Following Cleavage of the *Escherichia coli* Chromosome by EcoKI

**DOI:** 10.1371/journal.pone.0006542

**Published:** 2009-08-06

**Authors:** Laura Wardrope, Ewa Okely, David Leach

**Affiliations:** Institute of Cell Biology, University of Edinburgh, Edinburgh, United Kingdom; University of Massachusetts Medical School, United States of America

## Abstract

DNA double-strand breaks can be repaired by homologous recombination involving the formation and resolution of Holliday junctions. In *Escherichia coli*, the RuvABC resolvasome and the RecG branch-migration enzyme have been proposed to act in alternative pathways for the resolution of Holliday junctions. Here, we have studied the requirements for RuvABC and RecG in DNA double-strand break repair after cleavage of the *E. coli* chromosome by the EcoKI restriction enzyme. We show an asymmetry in the ability of RuvABC and RecG to deal with joint molecules *in vivo*. We detect linear DNA products compatible with the cleavage-ligation of Holliday junctions by the RuvABC pathway but not by the RecG pathway. Nevertheless we show that the XerCD-mediated pathway of chromosome dimer resolution is required for survival regardless of whether the RuvABC or the RecG pathway is active, suggesting that crossing-over is a common outcome irrespective of the pathway utilised. This poses a problem. How can cells resolve joint molecules, such as Holliday junctions, to generate crossover products without cleavage-ligation? We suggest that the mechanism of bacterial DNA replication provides an answer to this question and that RecG can facilitate replication through Holliday junctions.

## Introduction

Homologous recombination is used to repair DNA double-strand breaks in *E. coli*. This reaction is catalysed by RecBCD and RecA proteins, which resect DNA ends and mediate strand-exchange, respectively [1]. The products of strand exchange are understood to be joint molecules tethered to each other by Holliday junctions and replication forks. The Holliday junctions are then assumed to be migrated along the paired molecules by the RuvAB or RecG proteins and then resolved either by RuvC-mediated cleavage in the presence of RuvAB, followed by ligation, or in some unknown way in the presence of RecG [2]. Two main classes of hypotheses have been proposed to explain resolution of Holliday junctions by RecG. First, RecG could operate with an unknown nuclease to cleave Holliday junctions. A specific example of such a mechanism involving nicked Holliday junctions has been suggested based on a model proposed for *S. pombe* meiotic recombination [3]. Second, RecG could branch migrate one Holliday junction into a DNA end [4] or into another Holliday junction as originally hypothesised by Thaler and Stahl for lambda phage recombination [5]. Synthesis-dependent strand annealing (SDSA) is another example of this second class of cleavage-ligation independent model [6]. A unifying feature of these cleavage-ligation independent models is that they do not lead to crossing over. According to the first class of hypotheses, evidence of Holliday junction cleavage-ligation should be detected. According to the second class of hypotheses evidence for crossing over should not be detected. We have therefore set out to obtain evidence for Holliday junction cleavage-ligation and for crossing over via the RecG pathway. We see no evidence of Holliday junction cleavage-ligation but do detect resolution to crossover products implying that neither the first nor the second class of hypotheses is correct and requiring a new model for the action of RecG.

Previously, we developed a system for generating DNA double-strand breaks in the *E. coli* chromosome using the EcoKI restriction enzyme [7]. EcoKI is a type I restriction-modification complex that modifies hemimethylated DNA target sequences and cleaves fully unmethylated DNA target sequences. Its recognition sequence is AAC(N_6_)GTGC but cleavage occurs at a site distant from this sequence (reviewed in [8]. The restriction activity of EcoKI can be attenuated temporarily by the cell, a phenomenon referred to as restriction alleviation (RA). DNA damaging treatments that cause the formation of unmethylated target sites induce RA [9], [10], [11], [12]. RA is also observed when the genes encoding a restriction-modification system are transferred into an *E. coli* cell lacking that system. RA is dependent on the protease specified by the *clpX* and *clpP* genes [13]. ClpXP protease alleviates restriction by degrading the HsdR subunit of EcoKI as the complex translocates along the DNA [14]. ClpXP is also responsible for restriction alleviation of cells treated with UV light, naladixic acid or 2-aminopurine [14]. Notably, it has been proposed that the original function of RA lies in protecting the chromosome when recombination generates unmethylated target sequences [15]. We have used 2-aminopurine treatment of *clpX* mutant cells to generate DNA double-strand breaks and observe DNA repair by homologous recombination [7]. This system has features that distinguish it from other systems for studying DNA double-strand break repair. Because the breaks are generated by a restriction endonuclease, it is expected that the damage will be more uniform than the damage generated by a DNA damaging agent such as X- or γ-irradiation. However, in contrast to systems where a restriction endonuclease is induced in a cell, cleavage by EcoKI is expected on one sister chromosome only. Furthermore, since the cleaved target sequence is generated by DNA synthesis, the majority of cleaved sites are expected to lie in newly replicated DNA.

It was formerly reported that a *recG* mutant was highly sensitive to EcoKI mediated DNA cleavage while a *ruvABC* mutant was minimally sensitive [7]. However, further investigation revealed that several observations reported in that paper could not be reproduced. Notably, we were unable to reproduce the reported sensitivities of *recF*, *recJ*, *recQ* and *sbcC* strains, and were only able to detect a modest sensitivity of a *recN* strain. By contrast, significant sensitivity of a *ruvABC* mutant was detected and the sensitivities of *recA*, *recB* and *recG* mutants were confirmed [16]. The work reported here was designed to set the record straight with respect to the effects of the genes significantly implicated in the repair of EcoKI breaks and in particular to investigate the pathways of resolving recombination intermediates.

## Results

### Repair of DNA double-strand breaks is required for cell viability

Cromie and Leach reported that recombination defective mutants of Δ*clpX hsdR* ^+^ strains survive poorly following treatment with 2-aminopurine (2-AP; [7]. We have improved their method of analysis by treating cells with 2-AP at 20 µg/ml and following their survival as a function of time (Figure 1). Three rounds of replication are predicted to generate an unmethylated target: the first is required to incorporate 2-AP opposite cytosine, the second to incorporate thymine opposite 2-AP and the third to incorporate adenine opposite thymine. Consistent with the prediction that three rounds of DNA replication of about 30 minutes each are required to generate the unmethylated targets that are the substrates for cleavage by EcoKI, *recA*, Δ*recBCD*, Δ*recG* and Δ*ruvABC* mutants showed no decrease in viability after 50 minutes but were affected after 100 minutes of 2-AP treatment (Figure 1A). The kinetics of killing was similar in the *recA*, Δ*recG* and Δ*recBCD* mutant strains though the extent of killing was greater in Δ*recBCD*. Interestingly, the Δ*ruvABC* mutant showed continued killing at later times following treatment. On the other hand, the Δ*recG* Δ*ruvABC* strain was exquisitely sensitive to 2-AP treatment and already displayed killing at 50 minutes post treatment, suggesting a more rapid accumulation of unmethylated targets than the expected three rounds of DNA replication required in the other mutants. In all mutants apart from the Δ*recG* Δ*ruvABC* strain, there was little killing by 2-AP in an *hsdR* mutant strain (Figure 1B). The Δ*recG* Δ*ruvABC* strain showed some killing by 2-AP in the absence of EcoKI, but substantially less than in the presence of EcoKI. All together, these data indicate that the majority of killing after the 2-AP treatment was caused by the EcoKI endonuclease.

**Figure 1:** Sensitivity of recombination defective mutants to EcoKI breaks. Exponential cultures were treated with 20 µg/ml of 2-AP and relative viability calculated as described in Experimental Procedures. Error bars indicate 95% confidence intervals. (A) Indicated genotypes are in an *hsdR^+^ ΔclpX* background. The strains used were DL1902 (*rec^+^*), DL2656 (*recA*), DL1940 (*ΔrecG*), DL2659 (*ΔrecBCD*), DL1938 (*ΔruvABC*), DL 1962 (*ΔrecG ΔruvABC*). (B) Indicated genotypes are in an *hsdR514 ΔclpX* background. The strains used were DL1800 (*rec^+^*), DL2666 (*recA*), DL2133 (*ΔrecG*), DL2675 (*ΔrecBCD*), DL2114 (*ΔruvABC*), DL2667 (*recA ΔruvABC*), DL2671 (*recA ΔrecG*), DL2676 (*ΔrecBCD ΔruvABC*), DL2674 (*ΔrecBCD ΔrecG*), DL2149 (*ΔrecG ΔruvABC*). (C) Indicated genotypes are in an *hsdR^+^ ΔclpX* background. The strains used were DL1940 (*ΔrecG*), DL1938 (*ΔruvABC*), DL2656 (*recA*), DL2670 (*recA ΔrecG*), DL2657 (*recA ΔruvABC*).

The viability of different combinations of mutations was investigated to test the possible interactions between the “early” Δ*recA* mutation and the “late” Δ*recG* and Δ*ruvABC* mutations. As shown in Figure 1C, the sensitivity of a *recA* Δ*recG* double mutant strain to DNA double strand breaks induced by 2-AP was similar to the sensitivity of either *recA* or Δ*recG* single mutant strain suggesting that RecG and RecA may be operating in the same pathway. By contrast, the sensitivity of a Δ*ruvABC* mutant increased throughout the time course and at late times was greater than that of a *recA* mutant. At early times the sensitivity of a *recA* Δ*ruvABC* double mutant was greater than that of a Δ*ruvABC* mutant. These data suggest that at late times RuvABC contributes to a survival pathway independent of RecA and at early times RecA contributes to a survival pathway independent of RuvABC.

### *ruv* mutants accumulate Holliday junctions while *recG* mutants do not

To understand the role of RuvABC and RecG in processing branched DNA intermediates, we have carried out pulsed-field gel electrophoresis on the chromosomal DNA of Δ*clpX* mutants after treatment with 2-AP. The conditions used for gel electrophoresis allowed circular and branched molecules to be retained in the wells whereas linear DNA fragments of a wide spectrum of sizes (450 kb to 4.5 mb) migrated as a single band in the gel. As shown in Figures 2A1, treatment with 2-AP in the presence of EcoKI (*hsdR* ^+^ cells) induced the formation of linear DNA fragments above that observed in the absence of 2-AP (Figure 3A1) or the absence of EcoKI (Figure 3A2). Consistent with previous observations, Δ*recBCD* Δ*clpX* mutant strains treated with 2-AP in the presence of EcoKI accumulated more linear DNA [17], [18], [19], [20] and *recA* Δ*clpX* mutant strains treated with 2-AP in the presence of EcoKI showed loss of DNA from the wells, confirming the “reckless” DNA degradation previously observed in the absence of RecA after induction of DNA damage [21]. Surprisingly, the behaviours of Δ*recG* Δ*clpX* and Δ*ruv* Δ*clpX* mutants were very different from each other despite both mutants being sensitive to 2-AP. The Δ*recG* Δ*clpX* strain's response to 2-AP treatment was similar to the *rec^+^* Δ*clpX* strain whereas the Δ*ruvAB* Δ*clpX* and Δ*ruvC* Δ*clpX* strains showed no detectable linear DNA (Figure 2A1). Linear fragments were observed in the *recA* Δ*ruvAB* Δ*clpX*, *recA* Δ*ruvC* Δ*clpX*, Δ*recBCD* Δ*ruvAB* Δ*clpX and* Δ*recBCD* Δ*ruvC* Δ*clpX* mutant strains, suggesting that their absence in the Δ*ruvAB* Δ*clpX* and Δ*ruvC* Δ*clpX* mutant strains was caused by linear fragments trapped in the wells as they recombined with other DNA (Figure 2A1). To investigate if the lack of linear DNA in the Δ*ruvAB* Δ*clpX* and Δ*ruvC* Δ*clpX* strains was due to chromosomal fragments tied together by structures such as unresolved Holliday junctions, a plasmid expressing the bacteriophage resolvase RusA was introduced into these strains. As shown in Figures 2A2, the presence of a plasmid encoding the RusA nuclease liberated linear DNA from both Δ*ruv* Δ*clpX* strains; behaviour not observed in the presence of the plasmid vector lacking the *rusA* gene (Figure 2A3).

**Figure 2:** Pulsed field gel analysis of chromosomal DNA following treatment of Δ*clpX* mutant strains with 2-AP, prior to cleavage with *Not*I (A1, A2 and A3) and after cleavage with *Not*I (B1, B2 and B3). The *S. cerevisiae* chromosomes are shown in lane 1 as a molecular size standard, confirming the compression of linear fragments of 450 kb to 1.5 mb into a single band under the conditions used. This band of yeast chromosomes runs at the same position as linearized E.coli DNA (4.5 mb). (A1 and B1) Lanes 2–15, release of linear DNA into pulsed field gels from *rec* ^+^ and recombination defective strains: DL1902, DL2656, DL2659, DL3179, DL3184, DL2600, DL3201, DL3207, DL2670, DL3204, DL3208, DL2673, DL3200, DL3206. (A2 and B2) Lanes 2–15, release of linear DNA into pulsed field gels from *rec* ^+^ and recombination defective strains containing the plasmid pBAD-*rusA*: DL3122, DL3217, DL3123, DL3218, DL3219, DL3220, DL3221, DL3222, DL3223, DL3224, DL3225, DL3226, DL3227, DL3228. (A3 and B3) Lanes 2–15, release of linear DNA into pulsed field gels from *rec* ^+^ and recombination defective strains containing the plasmid pBAD18: DL3251, DL3252, DL3253, DL3254, DL3255, DL3256, DL3257, DL3258, DL3259, DL3260, DL3261, DL3262, DL3263, DL3264.

**Figure 3:** Pulsed field gel analysis of chromosomal DNA of Δ*clpX* mutant strains not exposed to EcoKI mediated DNA damage, prior to cleavage with *Not*I (A1, A2 and A3) and after cleavage with *Not*I (B1, B2 and B3). The *S. cerevisiae* chromosomes are shown in lane 1 as a molecular size standard, confirming the compression of linear fragments of 450 kb to 1.5 mb into a single band under the conditions used. This band of yeast chromosomes runs at the same position as linearized E.coli DNA (4.5 mb). (A1 and B1) Lanes 2–15, release of linear DNA into pulsed field gels from *rec* ^+^ and recombination defective strains – all strains are *hsdR* ^+^ and have not been treated with 2-AP: DL1902, DL2656, DL2659, DL3179, DL3184, DL2600, DL3201, DL3207, DL2670, DL3204, DL3208, DL2673, DL3200, DL3206. (A2 and B2) Lanes 2–15, release of linear DNA into pulsed field gels from *rec* ^+^ and recombination defective strains – all strains are *hsdR* ^−^ and have been treated with 2-AP: DL1800, DL2666, DL2675, DL3178, DL3180, DL2601, DL3203, DL3211, DL2671, DL3205, DL3210, DL2674, DL3202, DL3209. (A3 and B3) Lanes 2–15, release of linear DNA into pulsed field gels from *rec* ^+^ and recombination defective strains containing the plasmid pBAD-*rusA* – all strains are *hsdR* ^+^ and have not been treated with 2-AP: DL3122, DL3217, DL3123, DL3218, DL3219, DL3220, DL3221, DL3222, DL3223, DL3224, DL3225, DL3226, DL3227, DL3228.

The behaviour of these strains was further investigated by studying their chromosomal DNAs digested by the *Not*I restriction enzyme on pulsed field gels (Figures 2B1, 2B2 and 2B3) with respect to controls (Figures 3B1. 3B2 and 3B3). Strikingly, the deficit of *Not*I fragments entering the gel from 2-AP treated Δ*ruvAB* Δ*clpX* and Δ*ruvC* Δ*clpX* strains suggests that joint molecules were connecting a substantial proportion of *Not*I cleaved DNA. Following *Not*I cleavage, a small increase in linear fragment DNA entering the gel was observed in Δ*ruvAB* Δ*clpX* and Δ*ruvC* Δ*clpX* mutant strains over Δ*ruvAB recG* Δ*clpX* and Δ*ruvC* Δ*recG* Δ*clpX* mutant strains (Figure 2B1), which contrasts with the absence of fragments visualised in *ruv* and *ruv recG* mutants without *Not*I cleavage. This finding suggests that RecG is carrying out a role in resolving joint molecules in the absence of RuvABC but RecG is not as efficient in liberating *Not*I fragments as is RuvABC. Finally, the role of RecG requires chromosome fragmentation with *Not*I to be visualised, which is consistent with the products of RecG action not including linear molecules.

### Chromosome dimer resolution is required for cell viability in the presence and absence of RuvABC and RecG

In *E. coli*, crossing over can be assessed by its consequence on the segregation of the single circular chromosome [22]. Crossing over generates a single dimeric chromosomal structure, which is unable to segregate to the two daughter cells during cell division. Therefore, *E. coli* has evolved a dimer resolution pathway involving the XerCD proteins acting at the *dif* site, located close to the terminus of chromosome replication [23]. In *xerC*, *xerD* or *dif* mutants, dimers cannot be resolved back to monomers and the consequent segregation problem leads to cell death.

In order to test whether recombination stimulated by EcoKI cleavage of the chromosome results in crossover products leading to chromosome dimer formation, we studied the sensitivity of Δ*clpX* Δ*xerC* and Δ*clpX* Δ*dif* mutants to 2-AP in the presence or absence of Δ*ruvABC*, Δ*recG*, and *recA* (Figure 4). Δ*clpX* Δ*xerC* and Δ*clpX* Δ*dif* mutants were modestly sensitive to 2-AP (about 10 fold; Figure 4A). Δ*ruvABC* Δ*clpX* Δ*xerC* and Δ*ruvABC* Δ*clpX* Δ*dif* mutants were significantly more sensitive to 2-AP than Δ*ruvABC* Δ*clpX* mutants (about 100 fold; Figure 4B). Similarly, Δ*recG* Δ*clpX* Δ*xerC* and Δ*recG* Δ*clpX* Δ*dif* mutants were significantly more sensitive to 2-AP than Δ*recG* Δ*clpX* mutants (about 100 fold; Figure 4C). These results indicate that recombination in the presence or absence of RuvABC or RecG leads to the formation of a significant proportion of chromosome dimers that require XerCD action at *dif* for survival. Consistent with a requirement for recombination to produce dimers requiring XerCD and *dif* for resolution, a *recA* Δ*clpX* Δ*dif* strain was no more sensitive to 2-AP than a *recA* Δ*clpX* strain (Figure 4D).

**Figure 4:** Effect of *xerC* and *dif* mutations on cell sensitivity to EcoKI breaks. Exponential cultures were treated with 20 µg/ml of 2-AP and relative viability calculated as described in Experimental Procedures. Error bars indicate 95% confidence intervals. In addition to the genotypes shown, all strains carry the Δ*clpX* deletion. (A) Strains used were DL1902 (*rec^+^*), DL1930 (*rec^+^ xerC*), DL2245 (*rec^+^ dif*), DL1800 (*hsdR rec^+^*), DL2097 (*hsdR rec^+^ xerC*) and DL2244 (*hsdR rec^+^ dif*). (B) Strains used were DL1938 (Δ*ruvABC*), DL1952 (Δ*ruvABC xerC*), DL 2249 (Δ*ruvABC dif*), DL2114 (*hsdR ΔruvABC*), DL2118 (*hsdR ΔruvABC xerC*) and DL2248 (*hsdR ΔruvABC dif*). (C) Strains used were DL1940 (ΔrecG), DL1944 (ΔrecG *xerC*), DL2346 (Δ*recG dif*), DL2133 (*hsdR ΔrecG*), DL2136 (*hsdR ΔrecG xerC*) and DL2345 (*hsdR ΔrecG dif*). (D) Strains used were DL2656 (*recA*), DL2903 (*recA dif*), DL2666 (*hsdR recA*) and DL2904 (*hsdR recA dif*).

## Discussion

In this study, we have characterised the pathways of joint molecule resolution in *E. coli* following the generation of DSBs with EcoKI in a *clpX* mutant. Specifically, we have explored the roles of *ruvABC* and *recG* genes in the survival of EcoKI mediated DSBs, their roles in the formation of dimeric chromosomes and in resolving joint molecules detected on gels. Throughout this work, we have been careful to control for non-specific effects of 2-AP treatment by comparing the behaviour of *hsdR*+ and *hsdR* mutant strains. In all situations we attribute to double-strand break repair only the effects observed in the presence of EcoKI nuclease (*hsdR*+).

### Survival of cells after EcoKI-mediated DNA double-strand breaks

The *recA* and *recBCD* genes, essential for the early stages of DNA double-strand break repair (DSBR), are required for survival of breaks generated by EcoKI. In addition both the *recG* and *ruvABC* genes, responsible for the resolution of Holliday junctions, are required for survival, though a Δ*recG* Δ*ruvABC* double mutant is significantly more sensitive to these breaks than are the single mutants. The high sensitivity of the Δ*recG* Δ*ruvABC* double mutant may arise from a combination of factors. First, there is a notable sensitivity of this strain to 2-AP even in the absence of EcoKI. Second, the early response to 2-AP treatment suggests that, in this mutant, the pathway of DSB formation may be different to the other strains. Third, there may exist a pathway of survival (e.g. via replication fork reversal) that requires resolution of Holliday junctions even in the absence of recombination (see below). The observations that *recG* and *ruv* single mutants are sensitive to 2-AP is reminiscent of the requirements for both *recG* and *ruv* for the repair of SbcCD-induced breaks at a DNA palindrome [24]. Both of these reactions are predicted to be DSB repair events occurring following DNA replication between one cleaved and one intact sister chromosome.

Surprisingly, a *recA* mutant is not more sensitive than any other single mutant tested here and is less sensitive at late times than a Δ*ruvABC* mutant. This suggests the existence of a RecA-independent but RuvABC-dependent pathway for survival of double-strand breaks. The only known RuvABC-dependent, RecA-independent reaction is replication fork reversal (Seigneur et al. 1998) and it is possible that recovery of a small fraction of intact circular chromosomes could be mediated by a combination of RecBCD mediated degradation and RuvABC-mediated fork reversal as shown in Figure 5.

**Figure 5:** Illustration of how an intact monomeric circular chromosome might be generated without recombination following DNA double-strand breakage. In the absence of RecA, DSB repair would be prevented. Instead, a combination of replication fork reversal by RuvABC and DNA degradation by RecBCD could regenerate an intact circular chromosome and promote survival.

### Formation and resolution of Holliday junctions

In order to understand the contributions of RecG and RuvABC to the resolution of Holliday junctions, we analysed by pulsed field gel electrophoresis the genomic DNA of cells in which EcoKI breaks had been generated. Long linear DNA molecules are able to enter a pulsed field gel whereas long branched and circular molecules cannot (Nakayama et al., 1994). Because the *E. coli* chromosome is circular it does not enter the gel. As shown in Figure 2A1 and 2A3, linear DNA is generated by treatment of a Δ*clpX* mutant with 2-AP implying that cleavage with EcoKI produces some linear DNA fragments. Recombination of such linear fragments will produce branched molecules that will not enter the gel and, if these branched molecules include linear molecules joined together by Holliday junctions, cleavage-ligation of the junctions can regenerate linear DNA fragments (see Figure 6). Δ*ruvAB* Δ*clpX* and Δ*ruvC* Δ*clpX* mutants do not produce a detectable level of linear DNA, suggesting the presence of Holliday junctions tying DNA molecules together. Consistent with this explanation, expression of the bacteriophage resolvase RusA in the Δ*ruvAB* Δ*clpX* and Δ*ruvC* Δ*clpX* mutants liberates linear fragments (Figure 2A2). Surprisingly given its sensitivity to 2-AP, the DNA of a Δ*recG* Δ*clpX* mutant behaves similarly on a pulsed field gel to the DNA of a Δ*clpX* mutant following treatment with 2-AP. Within the limits of detection of this methodology, our data suggest that the RuvABC resolvase is able to act in the Δ*recG* Δ*clpX* mutant and resolve a substantial proportion of the Holliday junctions tying the DNA linear molecules together. Nevertheless, this action of RuvABC is not sufficient to prevent sensitivity of the Δ*recG* Δ*clpX* mutant to 2-AP. We suggest therefore, that the sensitivity of the Δ*recG* Δ*clpX* mutant to 2-AP is either explained by the presence of some critical unresolved joint molecules despite the ability of RuvABC to visibly resolve the Holliday junctions in our gel assay or by the action of RecG in a step other than the resolution of Holliday junctions.

**Figure 6:** Illustration of how linear DNA can be generated by cleavage-ligation or branch migration of Holliday junctions in the context of a circular chromosome. A. *cis* and *trans* configurations of DNA ends on a linear fragment are joined by an odd number of Holliday junctions. Cleavage-ligation of the junctions liberates the linear DNA. B. *cis* and *trans* configurations of DNA ends on a linear fragment are joined by an odd number of Holliday junctions. Branch migration will not liberate linear DNA. Instead it will convert an alpha-shaped molecule to a sigma-shaped molecule. C. *cis* and *trans* configurations of DNA ends on a linear fragment are joined by an even number of Holliday junctions. Cleavage-ligation of the junctions will liberate linear DNA. D. *cis* and *trans* configurations of DNA ends on a linear fragment are joined by an even number of Holliday junctions. Branch migration of the junctions will liberate linear DNA.

RecG and any proteins working with it are unable to produce a detectable level of linear DNA fragments in the absence of RuvABC (Figure 2A1 and 2A3). The generation of these fragments as a function of the presence of RuvABC, or RusA in the absence of RuvABC, suggests the junction of two DNA molecules by one or more Holliday junctions linking two DNA ends (Figure 6). Cleavage-ligation of Holliday junctions has the potential to generate linear DNA depending on the plane of resolution of the junctions and the number of junctions present (Figure 6A and 6C). Resolution can also occur by branch migration if the ends are joined by an even number of Holliday junctions (Figure 6D). However, resolution of junctions by branch migration will never generate linear DNA if the ends are joined by an odd number of junctions (Figure 6B). As observed in the *ruv* mutants, the RecG pathway does not result in linear DNA, which implies that no Holliday junction cleavage-ligation can be detected. If RecG can resolve joint molecules simply by branch migration, our result implies either that this reaction is too weak to liberate DNA fragments or that there are predominantly odd numbers of Holliday junctions between the DNA ends. Following cleavage with *Not*I, a small increase in the liberation of linear DNA fragments is observed in *ruv* mutants over what is observed in *ruv recG* mutants (Figure 2B1 and 2B3). This suggests that RecG is capable of resolving some joint molecules within the context of products that require *Not*I cleavage for visualisation. This is consistent with the proposal that RecG may resolve some critical junctions.

### Formation and resolution of chromosomal dimers

Mutations in *xerC* and *dif* confer modest sensitivity to EcoKI mediated breaks. This suggests that a proportion of these breaks are repaired by a mechanism that yields dimeric crossover products. Interestingly, Δ*xerC* and Δ*dif* mutations confer a greater sensitivity to EcoKI breaks in Δ*ruvABC* or Δ*recG* mutants. A similar sensitivity of both *recG* and *ruv* mutants to the inactivation of the XerCD/*dif* system has been observed after induction of DSBs using the rare-cutting endonuclease I-SceI [6]. The increase in sensitivity of the Δ*recG* mutant can be due to crossover products generated by cleavage-ligation of Holliday junctions using RuvABC. However, the reason for the increase in sensitivity of the Δ*ruvABC* mutant is not easy to explain, as no Holliday junction nuclease is known to act in conjunction with RecG and the pulsed field gel electrophoresis presented here shows that no cleavage-ligation of Holliday junctions can be detected in the presence of RecG and absence of RuvABC. The simplest implication of this work is that resolution of intermediates by RecG results in crossing over without cleavage-ligation of Holliday junctions.

### Conclusions

Here we show that, following induction of DNA double-strand breaks by EcoKI in a *clpX* mutant strain, RuvABC and RecG work very differently from each other and cannot be considered simply as catalysing steps in redundant pathways. RuvABC behaves as predicted for a protein that can resolve Holliday junctions by cleavage and this cleavage, followed by ligation, can lead to crossing over. Resolution by RecG also leads to crossing over but we can detect no evidence of Holliday junction cleavage-ligation via this pathway. This creates an apparent contradiction since all the standard cleavage-ligation independent models for recombination, such as SDSA, do not lead to crossing over.

A new model is required that can allow the maturation of a Holliday junction intermediate to a crossover product without junction cleavage-ligation. We suggest here that one way in which a Holliday junction can be matured to a crossover product without cleavage-ligation is if two new replication forks run through the junction. This would not be possible in most eukaryotic cells where new rounds of DNA replication are not initiated until after cell division. However, in bacteria new rounds of replication are normally initiated prior to cell division so it would be normal for an unresolved Holliday junction to act as a potential barrier to the passage of new forks. We suggest that RecG may facilitate the passage of the replication forks across the junction as detailed in Figure 7.

**Figure 7:** Model for the generation of chromosome dimers without Holliday junction cleavage-ligation. Bacteria, such as *E. coli*, have circular chromosomes and at normal growth rates reinitiate DNA replication before the previous round of replication has completed and before cell division takes place. This means that an unresolved Holliday junction is a potential barrier to the passage of the next set of replication forks. We propose here that replication through the Holliday junction may be possible and that this may be facilitated by the branch migration protein RecG. A. Chromosome in which a Holliday junction (HJ) has formed following the passage of a replication fork (RF1). A second pair of replication forks (RF2) are shown approaching the Holliday junction. The first two chromosomes to be produced by this replicating structure are labelled C1 and C2. The two chromosomes destined to be made from C1 are labelled C1.1 and C1.2 and the chromosomes destined to be made from C2 are labelled C2.1 and C2.2. The DNA strands that have exchanged to form the Holliday junction (and strands templated on these) are shown in red whereas the DNA strands that have not exchanged (and strands templated on these) are shown in blue. The four double-stranded molecules formed by the second pair of replication forks are shaded in light blue and pink. B. Two new forks (RF2) approaching the Holliday junction. When the pair of RF2 forks approaches the Holliday junction, the positive supercoiling ahead of the forks is predicted to push the junction ahead of them. At some point the forks are likely to stall, presumably because the Holliday junction impedes their progression. At this point, branch migration of the Holliday junction to the fork will lead to a swapping of newly synthesised sister chromosome arms. Chromosomes C1.1 and C2.1 will be connected to the unreplicated arm of C1 while chromosomes C1.2 and C2.2 will be connected to the unreplicated arm of C2. C. Formation of two monomeric and one dimeric chromosome. The replication machinery is reassembled on the two hybrid RF2 forks and replication continues. The figure illustrates the point where the RF2 forks have passed through the Holliday junction leaving the red strands crossed over (CO). The RF1 forks have completed their replication and no longer exist. When the RF2 forks complete replication and meet at the terminus, two monomeic blue chromosomes (C1.1 and C2.2) will have formed as well as one dimeric red (crossover) chromosome (C1.2–C2.1). The shading of the molecules formed by the RF2 replication forks illustrates that the red double strands are crossed over whereas the blue double strands are not.

## Materials and Methods

### Bacterial strains

All the *E. coli* strains described in Table 1 are derivatives of BW27784 with the following genotype: *lacI* ^q^, *rrnB3*, Δ*lacZ4787*, *hsdR514*, Δ*araBAD567*, Δ*araFGH*, Δ*rhaBAD568*, Φ(Δ*araEp*P_CR18_-*araE*) [25]. This strain allows homogeneous expression from the P*_BAD_* promoter thanks to a deletion of the genes encoding the AraFGH transporter and expression of the low-affinity, high-capacity AraE transporter from the constitutive promoter P_CP18_.

**Table 1:** Bacterial Strains.

Strain Number	Relevant Genotype
DL1800	Δ*clpX_1789_ hsdR514*
DL1902	Δ*clpX_1789_*
DL1930	Δ*clpX_1789_ xerC*_Y17_::*cat*
DL1938	Δ*clpX_1789_ ΔruvABC*_65_ *eda*_51_::Tn*10*
DL1940	Δ*clpX_1789_ ΔrecG_263_::kan*
DL1944	Δ*clpX_1789_ xerC*_Y17_::*cat ΔrecG*_263_::*kan*
DL1952	Δ*clpX_1789_ xerC*_Y17_::*cat ΔruvABC*_65_ *eda*_51_::Tn*10*
DL1962	Δ*clpX_1789_ ΔrecG*_263_::*kan ΔruvABC*_65_ *eda*_51_::Tn*10*
DL2097	Δ*clpX_1789_ hsdR514 xerC*_Y17_::*cat*
DL2114	Δ*clpX_1789_ hsdR514 ΔruvABC*_65_ *eda*_51_::Tn*10*
DL2118	Δ*clpX_1789_ hsdR514 xerC*_Y17_::*cat ΔruvABC*_65_ *eda*_51_::Tn*10*
DL2133	Δ*clpX_1789_ hsdR514 ΔrecG*_263_::*kan*
DL2136	Δ*clpX_1789_ hsdR514 xerC*_Y17_::*cat ΔrecG*_263_::*kan*
DL2149	Δ*clpX_1789_ hsdR514 ΔrecG*_263_::*kan ΔruvABC*_65_ *eda*_51_::Tn*10*
DL2244	Δ*clpX_1789_ hsdR514 difΔ*6::*kan*
DL2245	Δ*clpX_1789_ difΔ*6::*kan*
DL2248	Δ*clpX_1789_ hsdR514 difΔ*6::*kan ΔruvABC*_65_ *eda*_51_::Tn*10*
DL2249	Δ*clpX_1789_ difΔ*6::*kan ΔruvABC*_65_ *eda*_51_::Tn*10*
DL2345	Δ*clpX_1789_ hsdR514 difΔ*6::*kan ΔrecG*_265_::*cat*
DL2346	Δ*clpX_1789_ difΔ*6::*kan ΔrecG*_265_::*cat*
DL2600	Δ*clpX_1789_ ΔrecG_2472_*
DL2601	Δ*clpX_1789_ hsdR514 ΔrecG_2472_*
DL2656	Δ*clpX_1789_ recA*::*cat*
DL2657	Δ*clpX_1789_ ΔruvABC*_65_ *eda*_51_::Tn*10 recA*::*cat*
DL2659	Δ*clpX_1789_ ΔrecBCD*::*kan*
DL2661	Δ*clpX_1789_ ΔruvABC*_65_ *eda*_51_::Tn*10 ΔrecBCD*::*kan*
DL2666	Δ*clpX_1789_ hsdR514 recA*::*cat*
DL2667	Δ*clpX_1789_ hsdR514 ΔruvABC*_65_ *eda*_51_::Tn*10 recA*::*cat*
DL2670	Δ*clpX_1789_ ΔrecG_2472_ recA*::*cat*
DL2671	Δ*clpX_1789_ hsdR514 ΔrecG_2472_ recA*::*cat*
DL2673	Δ*clpX_1789_ ΔrecG_2472_ ΔrecBCD*::*kan*
DL2674	Δ*clpX_1789_ hsdR514 ΔrecG_2472_ ΔrecBCD*::*kan*
DL2675	Δ*clpX_1789_ hsdR514 ΔrecBCD*::*kan*
DL2676	Δ*clpX_1789_ hsdR514 ΔruvABC*_65_ *eda*_51_::Tn*10 ΔrecBCD*::*kan*
DL2903	Δ*clpX_1789_ difΔ*6::*kan recA*::*cat*
DL2904	Δ*clpX_1789_ hsdR514 difΔ*6::*kan recA*::*cat*
DL3122	Δ*clpX_1789_*, pBAD-*rusA*
DL3123	Δ*clpX_1789_ ΔrecBCD*::*kan*, pBAD-*rusA*
DL3178	Δ*clpX_1789_ hsdR514 ΔruvAB_2757_*
DL3179	Δ*clpX_1789_ ΔruvAB_2757_*
DL3180	Δ*clpX_1789_ hsdR514 ΔruvC_2731_*
DL3184	Δ*clpX_1789_ ΔruvC_2731_*
DL3200	Δ*clpX_1789_ ΔruvAB_2757_ ΔrecG*_263_::*kan*
DL3201	Δ*clpX_1789_ ΔruvAB_2757_ recA*::*cat*
DL3202	Δ*clpX_1789_ hsdR514 ΔruvAB_2757_ ΔrecG*_263_::*kan*
DL3203	Δ*clpX_1789_ hsdR514 ΔruvAB_2757_ recA*::*cat*
DL3204	Δ*clpX_1789_ ΔruvAB_2757_ ΔrecBCD*::*kan*
DL3205	Δ*clpX_1789_ hsdR514 ΔruvAB_2757_ ΔrecBCD*::*kan*
DL3206	Δ*clpX_1789_ ΔruvC_2731_ ΔrecG*_263_::*kan*
DL3207	Δ*clpX_1789_ ΔruvC_2731_ recA*::*cat*
DL3208	Δ*clpX_1789_ ΔruvC_2731_ ΔrecBCD*::*kan*
DL3209	Δ*clpX_1789_ hsdR514 ΔruvC_2731_ ΔrecG*_263_::*kan*
DL3210	Δ*clpX_1789_ hsdR514 ΔruvC_2731_ ΔrecBCD*::*kan*
DL3211	Δ*clpX_1789_ hsdR514 ΔruvC_2731_ recA*::*cat*
DL3217	Δ*clpX_1789_ recA*::*cat*, pBAD-*rusA*
DL3218	Δ*clpX_1789_ ΔruvAB_2757_*, pBAD-*rusA*
DL3219	Δ*clpX_1789_ ΔruvC_2731_*, pBAD-*rusA*
DL3220	Δ*clpX_1789_ ΔrecG_2472_*, pBAD-*rusA*
DL3221	Δ*clpX_1789_ recA*::*cat ΔruvAB_2757_*, pBAD-*rusA*
DL3222	Δ*clpX_1789_ recA*::*cat ΔruvC_2731_*, pBAD-*rusA*
DL3223	Δ*clpX_1789_ recA*::*cat ΔrecG_2472_*, pBAD-*rusA*
DL3224	Δ*clpX_1789_ ΔrecBCD*::*kan ΔruvAB_2757_*, pBAD-*rusA*
DL3225	Δ*clpX_1789_ ΔrecBCD*::*kan ΔruvC_2731_*, pBAD-*rusA*
DL3226	Δ*clpX_1789_ ΔrecBCD*::*kan ΔrecG_2472_*, pBAD-*rusA*
DL3227	Δ*clpX_1789_ ΔruvAB ΔrecG*_263_::*kan*, pBAD-*rusA*
DL3228	Δ*clpX_1789_ ΔruvC ΔrecG*_263_::*kan*, pBAD-*rusA*
DL3251	Δ*clpX_1789_*, pBAD18
DL3252	Δ*clpX_1789_ recA*::*cat*, pBAD18
DL3253	Δ*clpX_1789_ ΔrecBCD*::*kan*, pBAD18
DL3254	Δ*clpX_1789_ ΔruvAB_2757_*, pBAD18
DL3255	Δ*clpX_1789_ ΔruvC_2731_*, pBAD18
DL3256	Δ*clpX_1789_ ΔrecG_2472_*, pBAD18
DL3257	Δ*clpX_1789_ recA*::*cat ΔruvAB_2757_*, pBAD18
DL3258	Δ*clpX_1789_ recA*::*cat ΔruvC_2731_*, pBAD18
DL3259	Δ*clpX_1789_ recA*::*cat ΔrecG_2472_*, pBAD18
DL3260	Δ*clpX_1789_ ΔrecBCD*::*kan ΔruvAB_2757_*, pBAD18
DL3261	Δ*clpX_1789_ ΔrecBCD*::*kan ΔruvC_2731_*, pBAD18
DL3262	Δ*clpX_1789_ ΔrecBCD*::*kan ΔrecG_2472_*, pBAD18
DL3263	Δ*clpX_1789_ ΔruvAB ΔrecG*_263_::*kan*, pBAD18
DL3264	Δ*clpX_1789_ ΔruvC ΔrecG*_263_::*kan*, pBAD18

The *ΔclpX_1789_, ΔrecG_2472_, ΔruvAB_2757_*, and *ΔruvC_2731_* mutations were generated by plasmid-mediated gene replacement (PMGR) using pTOF24 derivative vectors, carrying homology arms spanning the gene of interest [26]. These homology arms were generated by crossover PCR using primers described in Table 2 and inserted into pTOF24 using *Sal*I and *Pst*I restriction enzymes. The mutations *xerC*_Y17_::*cat* (derived from strain DS984 obtained from D. Sherratt), *ΔruvABC*_65_ *eda*_51_::Tn10 (derived from strain N4155 obtained from R. Lloyd), *ΔrecG*_263_::*kan* (derived from strain N3793 obtained from R. Lloyd), *difΔ*6::*kan* (derived from strain GR47 obtained from D. Sherratt), *recA*::*cat* (derived from strain DB1318 obtained from D. Botstein) and *ΔrecBCD*::*kan* (derived from strain JJC1086 obtained from B. Michel) were introduced by P1 transduction. *HsdR* ^+^ derivatives were made by bacteriophage λ insertion and excision as described by Arber and collaborators [27] using λ NM1048 containing the wild type *hsdR* gene [28]. The HsdR phenotype was tested using methylated and unmethylated derivatives of λ clear and λ virulent. The plasmids pBAD18 [29] and its derivative pBAD-*rusA*, constructed by V. Bidnenko, were obtained from B. Michel.

**Table 2:** Restriction enzyme sites are underlined and the complementary parts of the primers useful for the crossover strategy are shown in bold.

Name	Primer sequence 5′ to 3′	Use
Δ*clpX*-F1	AAAAAGTCGACGCAGGGGCAAAAGGTAAAC	Crossover PCR to make Δ*clpX_1789_* K.O. fragment for pTOFΔ*clpX* construction
Δ*clpX*-R1	**CGACGTCTTCCATTTGCCTGAGCC** ATCTTTG	
Δ*clpX*-F2	**GGCTCAGGCAAATGGAAGACGTCG** AAAAAGTGG	
Δ*clpX*-R2	AAAAACTGCAGCGCTTCCAGACAACGGATAG	
Δ*recG*-F1	AAAAAGTCGACGCATTTTGATGGGACAGGAG	Crossover PCR to make Δ*recG_2472_* K.O. fragment for pTOFΔ*recG* construction
Δ*recG*-R1	**GTAACGTTCCGTGTTACTAAGTGC** TGCGCCAAC	
Δ*recG*-F2	**GCACTTAGTAACACGGAACGTTAC** TCGAATGC	
Δ*recG*-R2	AAAAACTGCAGATGGGCAAAAACTACGATGC	
Δ*ruvAB*-F1	AAAAACTGCAGGATCCCGACGTGATTACTCC	Crossover PCR to make Δ*ruvAB_2757_* K.O. fragment for pTOFΔ*ruvAB* construction
Δ*ruvAB*-R1	**TTACGGCATTTCGATGATGCCTCT** GAGTCTGC	
Δ*ruvAB*-F2	**AGAGGCATCATCGAAATGCCGTAA** GTCGGATTG	
Δ*ruvAB-*R2	AAAAAGTCGACTGACGATTGGTGTAGCGATG	
Δ*ruvC*-F1	AAAAACTGCAGATGGTTCCGTTGCCTATCTG	Crossover PCR to make Δ*ruvC_2731_* K.O. fragment for pTOFΔ*ruvC* construction
Δ*ruvC*-R1	**TCGCATTCTGACTAATAGCCATCA** CGCGTCTC	
Δ*ruvC*-F2	**TGATGGCTATTAGTCAGAATGCGA** TGCAGATG	
Δ*ruvC*-R2	AAAAAGTCGACGGCTGACAGAACGACAAAAAC	

### Standard DSBR assay

This assay was used to obtain the viability curves presented in Figures 1 and 2. An overnight culture in LB at 37°C was diluted in triplicate to an optical density (O.D.) of A_600_ = 0.02 and cultured to an O.D. of 0.2 in LB at 37°C under agitation. The three cultures were diluted to an O.D. of 0.02 in LB and grown at 37°C to an O.D. of 0.1 where they were split and 20 µg/ml of 2-AP was added to one flask of each culture. A sample of each culture was taken, diluted appropriately in LB and plated in triplicate onto L agar plates. The six cultures were incubated under agitation at 37°C and samples from each flask were taken every 50 minutes for 250 minutes. At each time point, samples were diluted appropriately before plating in triplicate on L agar plates and O.D. measurements were taken. Plates were incubated overnight at 37°C and the resulting colonies counted to give an indication of viable cells/ml. Relative viability was calculated as the viability of cells grown in the presence of 2-AP divided by the viability of cells grown in the absence of 2-AP. At least two independent assays were carried out for each strain and the graphs presented show the results of the combined independent experiments. The concentration of 2-AP used was based on the titrations carried out by Cromie and Leach [7] and 20 µg/ml was chosen as a minimal concentration at which clear effects on viability could be observed.

### Pulsed field gel electrophoresis (PFGE)

Overnight cultures grown in LB at 37°C of strains to be tested were diluted to an O.D. of A_600_ = 0.02 in LB and grown to O.D. 0.2 at 37°C under agitation. At that time, when appropriate, 100 µg/ml of 2-AP was added and the cultures were incubated for a further 2.5 hours (strains carrying the pBAD-*rusA* plasmid were always cultured in the presence of 0.002% arabinose to induce expression of RusA). At this point, 5 ml samples of cultures were extracted and spun down for 10 minutes at 3,500 rpm before resuspending the pellet in TEE solution (10 mM Tris, 100 mM EDTA, 100 mM EGTA, pH 8.5) to give an O.D. of 0.9. 350 µl of cells was mixed with 350 µl of 2% low melting point agarose (GIBCO) and cooled to 55°C. The mixture was immediately pipetted into disposable Biorad CHEF plug moulds and refrigerated until set. The plugs were then removed from the moulds and each set of ten incubated in 10 ml of lysozyme solution at 37°C with gentle agitation for two hours. Plugs were incubated overnight at 55°C in 5 ml of proteinase K solution and then rinsed in 10 ml TE buffer (10 mM Tris, 1 mM EDTA, pH 7.5) for 3X 1 hour. Plugs were then washed in 10 ml 1mM PMSF solution in TE buffer for 2 X 1 hour and then rinsed in 10 ml TE buffer for 2X 30 minutes. All TE and PMSF wash steps were carried out at room temperature under gentle agitation. The plugs were stored in TE buffer at 4°C and used within two months. The gels presented are representative of at least two gels run using plugs prepared from at least two independent cultures. In these experiments a concentration of 100 µg/ml 2-AP was used to ensure visualisation of chromosome fragmentation in the light of the experience of Cromie and Leach [7].

When agarose embedded DNA was required to be digested by *Not*I, single plugs were equilibrated in 1 ml of the appropriate 1X restriction buffer for one hour at room temperature. Then, the buffer was replaced with 350 µl reaction buffer containing 30–50 units of restriction enzyme and incubated for 4 hours at 37°C. Following digestion, plugs were used immediately for PFGE.

Plugs were halved and placed on the comb of the PFG apparatus. 100 ml of 1% (w/v) high-strength agarose (AquaPor™) was made up fresh in 0.5X TBE and cooled to 55°C. 0.5 µg/ml of ethidium bromide was added and the agarose carefully poured around the plugs attached to the comb. The gel was left to set at 4°C and the same agarose solution used to pour the gel was pipetted into the gaps left by the comb. The gel was run in 0.5X TBE using CHEF-DR™ II (Biorad) PFGE equipment. PFGE was carried out using the following parameters: initial switch time 5 seconds; final switch time 30 seconds; run time 17 hours; voltage 5 V/cm and temperature 4°C. Gels were viewed using a UV trans-illuminator.
